The article "Antileukemic Effects of Anti-miR-146a, Anti-miR-155, Anti-miR-181a, and Prednisolone on Childhood Acute Lymphoblastic Leukemia" was retracted in 2024. Reasons: signs of a paper mill; compromised peer review; unreliable results or conclusions.

# Antileukemic Effects of Anti-miR-146a, Anti-miR-155, Anti-miR-181a, and Prednisolone on Childhood Acute Lymphoblastic Leukemia

**DOI:** 10.1155/2021/3207328

**Published:** 2021-11-28

**Authors:** Burak Durmaz, Bakiye Goker Bagca, Ozgur Cogulu, Sunde Yilmaz Susluer, Araz Alpay, Serap Aksoylar, Cumhur Gunduz

**Affiliations:** ^1^Ege University, Faculty of Medicine, Department of Medical Genetics, 35100, Bornova, Izmir, Turkey; ^2^Aydin Adnan Menderes University, Faculty of Medicine, Department of Medical Biology, 09100 Aydin, Turkey; ^3^Ege University, Faculty of Medicine, Department of Pediatrics, 35100, Bornova, Izmir, Turkey; ^4^Ege University, Faculty of Medicine, Department of Medical Biology, 35100, Bornova, Izmir, Turkey; ^5^Ege University, Institute of Health Sciences, 35100, Bornova, Izmir, Turkey

## Abstract

Prednisolone has been used frequently in the treatment of acute lymphoblastic leukemia. However, to overcome the challenges of the treatment, the development of additional therapies is of great importance. Small, non-protein-coding RNAs, namely, microRNAs (miRNAs), are critical epigenetic regulators with physiological and pathological importance. This study is aimed at determining the effects of miR-146a, miR-155, and miR-181a inhibition with their corresponding anti-miRs on both leukemic and healthy cells, individually and with prednisolone. Leukemic (SUP-B15) and healthy B-lymphocyte (NCI-BL 2171) cell lines were used in this study. A total of 12 experimental groups included individual and combinational silenced ALL-associated miRNAs (hsa-miR-155, hsa-miR-146a, and hsa-miR-181a) and their combination with prednisolone. Cytotoxicity, proliferation, cell cycle, and apoptosis analyses were performed by using WST-1, trypan blue, APC-BrdU, Annexin V, and JC-1 methods in each study group, respectively. To control the effectiveness of anti-miR transfection and prednisolone application, miRNA expression analysis was performed from all groups. Anti-miR application was effective on the viability, proliferation, cell cycle, and apoptosis of leukemia cells, and this effect was increased with prednisolone administration. In addition, this activity was found to be very low on healthy cells. In conclusion, anti-miR applications may have the potential for clinical use of adjuvant to or as an alternative to conventional therapies for childhood acute lymphoblastic leukemia.

## 1. Introduction

Acute lymphoblastic leukemia (ALL) is a hematological malignancy originating from the disruption in the genetic structure of a single lymphoid precursor/progenitor cell. Although it is classified as B- or T-cell ALL according to the cell type they originate from, it is also grouped as adult or childhood ALL according to the age of onset. It is known as one of the most common cancers in childhood [1]. Prednisolone is a glucocorticoid approved by the FDA for the treatment of acute leukemias in the mid-1950s. It is the primary agent used in the treatment of ALL and has remained an essential component of therapy together with other chemotherapeutics. Its cytotoxic effect is mediated through the binding of glucocorticoid receptors which then repress the activity of transcription factors such as activating protein-1 or nuclear factor-*κ*B thus inhibiting cytokine production, altering the expression of various oncogenes, and inducing apoptosis [2]. Although ALL is revealed to be the most successful treatment model in pediatric cancer medicine as the significant survival rate improvement to >90% today, relapse and drug resistance remain to be significant subjects [3]. To overcome the challenges of the treatment such as recurrence or drug resistance, developing novel targeted therapies have great importance in addition to prednisolone treatment [4]. MicroRNAs (miRNA) are the most important epigenetic regulators, which do not encode a protein and provide posttranscriptional regulation of the genes. It has been associated with both physiological and pathological processes by regulating gene expression by degrading mRNAs or suppressing protein synthesis. Since the early 2000s, they have played an important role in molecular research because of their potential roles in cancer treatment [5]. The miRNAs selected for this study, namely, hsa-miR-146a, hsa-miR-155, and hsa-miR-181a are parts of the microRNAs in the cancer pathway [6]. Upregulated miR-146a, miR-155, and miR-181a levels are also described particularly in ALL progression [7–9]. Differentially expressed miRNAs are revealed to be important in the initiation and progression of ALL. As shown in various studies, these miRNAs can be used as noninvasive diagnostic and prognostic biomarkers in the monitoring early stages of ALL, accurate classification of different molecular subgroups, and identification of novel therapeutic agents [10].

The article "Antileukemic Effects of Anti-miR-146a, Anti-miR-155, Anti-miR-181a, and Prednisolone on Childhood Acute Lymphoblastic Leukemia" was retracted in 2024. Reasons: signs of a paper mill; compromised peer review; unreliable results or conclusions.

In addition, our previously published research revealed that a dramatic reduction in the expression levels of the mentioned miRNAs, following the treatment, highlights these miRNAs as an attractive target for ALL studies [9]. Therefore, in this study, we aimed to determine the possible antileukemic effects of miR-146a, miR-155, and miR-181a by inhibiting them with their relevant anti-miRs and investigate the possible effects in combination with conventional prednisolone application.

## 2. Materials and Methods

### 2.1. Cell Culture

The acute lymphoblastic leukemia cell line SUP-B15 (ATCC, CRL-1929) and healthy B-lymphocyte cell line NCI-BL 2171 (ATCC, CRL-5969) were commercially obtained. The SUP-B15 and NCI-BL 2171 cells were cultured in IMDM (Gibco, Cat. No: 12440053) and RPMI 1640 (Gibco, Cat. No: 11875085) mediums supplemented with 2 mM L-glutamine, 1% penicillin-streptomycin, and 10% FBS, respectively, in a cell culture incubator (Thermo Electron Corporation's Class 100) at 37°C, 95% humidity, and 5% CO_2_. Light (Olympus-CH30) and inverted (Olympus-CKX41) microscopy were used to observe the viability and proliferation of the cells. The cell maintenance and all experiments were performed in an ultraviolet-sterilized laminar airflow cabinet (ESCO Class II, Biological Safety Cabinets).

### 2.2. Chemical Agent Preparation

Methylprednisolone (lyophilized, MW: 496.532 g/mol) was dissolved in 2135 *μ*l ddH_2_O to adjust the final concentration of 50 mM.

### 2.3. Experimental Design

Experimental groups that included individual and combinational silenced ALL-associated miRNAs (hsa-miR-146a, hsa-miR-155, hsa-miR-181a, and hsa-let-7a as control) and their combination with prednisolone were designed (Table 1). A total of 12 groups were structured concerning the study design.

### 2.4. Cytotoxicity Assay

The cytotoxic effect of prednisolone on the acute lymphoblastic leukemia cell line SUP-B15 and healthy B-lymphocyte cell line NCI-BL 2171 was evaluated in a time- and dose-dependent manner by using colorimetric WST-1 (Cell Biolabs, Cat. No: CBA-253) assay in triplicate for each time and dose group. The SUP-B15 and NCI-BL 2171 cells were seeded into each well of a 96-well plate at the 2.5 × 10^5^ and 6 × 10^5^ cells/ml concentration, respectively. Prednisolone was treated in the cells at the dose range between 100 nM and 100 *μ*M at 50 *μ*l volume, and the final volume of each well reached 100 *μ*l. Untreated cells were used as the control group. After 24, 48, and 72 h incubation periods, 10 *μ*l WST-1 solution was added into each well, and formazan transformation was measured at 450 nm and 620 nm wavelengths in the Multiskan FC microplate reader (Thermo Scientific, Multiskan FC, Finland) in every 15 min. IC_50_ values of prednisolone were calculated by GraphPad Prism 6.0 (GraphPad software).

### 2.5. Anti-miR Transfection

SUP-B15 and NCI-BL 2171 cells were seeded in 6-well plates sufficient for all experimental groups, with a final concentration of 5 × 10^5^ cells/1.5 ml Opti-MEM medium (Gibco, Cat. No: 11058-021). The transfection agents were prepared using a 9 *μ*l Lipofectamine RNAiMAX reagent (Life Technologies, Cat. No: 13778-150), 150 *μ*l Opti-MEM medium required for each transfection process. Each mirVana miRNA inhibitor (anti-hsa-miR-146a, anti-hsa-miR-155, anti-hsa-miR-181a, and anti-hsa-let-7a; Thermo Fisher Scientific, Cat. No: 4464084) was prepared in an amount sufficient for all experiments using 150 *μ*l Opti-MEM medium with a final concentration of 30 pmol. The transfection agent and the anti-miRs were mixed in a 1 : 1 volume ratio and incubated for 5 min at room temperature. Afterward, 300 *μ*l of this mixture was added to the appropriate groups. In groups without transfection, 300 *μ*l of Opti-MEM medium was added to keep concentrations constant.

The article "Antileukemic Effects of Anti-miR-146a, Anti-miR-155, Anti-miR-181a, and Prednisolone on Childhood Acute Lymphoblastic Leukemia" was retracted in 2024. Reasons: signs of a paper mill; compromised peer review; unreliable results or conclusions.

### 2.6. Prednisolone Treatment

The groups which will be treated by IC_50_ dose of prednisolone were added 200 *μ*l prednisolone dissolved in Opti-MEM medium in proper concentration. In groups without prednisolone, 200 *μ*l of Opti-MEM medium was added to keep concentrations constant.

### 2.7. miRNA Expression Analysis

To control the effectiveness of anti-miR transfection, miRNA isolation from all groups was performed using the mirVana miRNA Isolation Kit (Thermo Fisher, Cat. No: AM1561) after the 48^th^ hour of the application period. Measuring the concentrations and purity of the isolated RNA samples was carried out using NanoDrop 1000 (Thermo Scientific) device and software. Synthesis of cDNA from samples with appropriate purity and quantity was performed using the TaqMan miRNA Reverse Transcription Kit (Cat. No: 4366596). RT-qPCR was carried out using TaqMan Advanced miRNA Assays (hsa-miR-155, hsa-miR-146a, hsa-miR-181a, and hsa-let-7a; Thermo Fisher Scientific, Cat. No: A25576; (Table 2), TaqMan Universal PCR Master Mix (Applied Biosystems, Cat. No: 4304437), and Applied Biosystems 7500 fast real-time PCR instrument.

### 2.8. Cell Viability Assay

Viability and proliferation analyses were determined at 48^th^ hour after anti-miR and prednisolone treatment using trypan blue 0.4% (Invitrogen, Cat. No: T10282) and light microscopy (Olympus-CH30).

### 2.9. Cell Cycle Analysis

The effects of the anti-miR and prednisolone of the cell cycle were determined at 48^th^ hour using the BrdU (Thermo Fisher, Cat No: B23151) method according to manufacturer's instructions, and the results were evaluated using Bd Accuri C6 (BD Biosciences Pharmingen) flow cytometry at FL3 (7-AAD-A) and FL4 (BrdU-APC A) channels.

### 2.10. Apoptosis Analysis

Apoptosis analyses were performed at the 48^th^ hour after anti-miR and prednisolone treatment by using Annexin V (BD Pharmingen, Cat. No: 556547) and MitoScreen JC-1 (BD Pharmingen, Cat. No: 551302) according to manufacturer's instructions. In addition, mitochondrial membrane potential changes were also detected by MitoScreen JC-1 assay. The results were evaluated by Bd Accuri C6 (BD Biosciences Pharmingen) flow cytometry.

The article "Antileukemic Effects of Anti-miR-146a, Anti-miR-155, Anti-miR-181a, and Prednisolone on Childhood Acute Lymphoblastic Leukemia" was retracted in 2024. Reasons: signs of a paper mill; compromised peer review; unreliable results or conclusions.

### 2.11. Statistical Analysis

IC_50_ dose of the prednisolone was calculated using a nonlinear regression log (inhibitor) vs. normalized response. Categorical variables were given as percentages and fold changes. The comparison of the groups was carried out with Fisher's exact probability test. Statistical analyses were made with GraphPad Prism 5.0 (GraphPad Software, Inc.), and significance was taken as *p* < 0.05.

## 3. Results

### 3.1. Prednisolone Has a Cytotoxic Effect on Acute Lymphoblastic Leukemia Cells at Lower Concentrations but Not on Healthy B-Lymphocyte Cells

The IC_50_ values of the prednisolone for the SUP-B15 and NCI-BL 2171 cell lines were determined as 20.20 *μ*M (*r*^2^ = 0.97) and 916.3 *μ*M (*r*^2^ = 0.98) at the 48^th^ hour, respectively (Figure 1).

### 3.2. Anti-miR Treatment Enhances the Cytotoxic Effect of Prednisolone on Leukemia Cells but It Is Ineffective on B-Lymphocytes

The effectiveness of the anti-miR transfection was validated by RT-qPCR (Supplementary Figure 1). All anti-miR treatments significantly enhanced the cytotoxic effect of the prednisolone on leukemia cells (mean 15.13%, max. value 55.00%, min. value 0.00%, *p* < 0.05; Table 3, Figure 2). It was determined that there were no living cells in the anti-miR-146a + anti-miR-155 + anti-miR-181a + anti-let-7e combination and prednisolone-treated group (viability percentage 0.00%, *p* < 0.0001). On the other hand, anti-miR treatment did not show a distinct effect on the cytotoxic effect of the prednisolone on healthy cells. The viability percentage of the cells was approximately 50% (mean 50.88%, max. value 58.18%, min. value 41.10%, *p* < 0.05).

### 3.3. The Anti-miR and Prednisolone Treatment Affects Leukemia Cell Cycle

The treatments did not cause a change in the cell accumulation level in the G0/G1 phase of SUP-B15 childhood ALL cells compared to the control group (control 56.03%, mean 66.38%, max. value 75.58%, min. value 49.68%, *p* > 0.05). G2/M phase accumulation of SUP-B15 childhood ALL cells was not changed compared to the control group (control 29.04%, mean 29.55%, max. value 49.68%, min. value 18.75%, *p* < 0.05). All treatment groups decreased S phase accumulation compared to the control group (control 14.93%, mean 4.07%, max. value 11.96%, min. value 0.47%, *p* > 0.05). It has been determined that the treatments did not cause a distinct change in the cell cycle of NCI-BL 2171 healthy B-lymphocytes (G0/G1 phase control 40.64%, mean 56.45%; S phase control 21.93%, mean 21.22%; G2/M phase control 37.43%, mean 22.33%; *p* > 0.05; Table 4, Figures 3(a) and 3(b), Supplementary Figure 2).

The article "Antileukemic Effects of Anti-miR-146a, Anti-miR-155, Anti-miR-181a, and Prednisolone on Childhood Acute Lymphoblastic Leukemia" was retracted in 2024. Reasons: signs of a paper mill; compromised peer review; unreliable results or conclusions.

### 3.4. The Anti-miR Combination Improves Apoptotic Effects of Prednisolone on Leukemic Cells

According to Annexin V results, prednisolone induced apoptosis 32.30 folds compared to controls in ALL cells (*p* < 0.0001). Although anti-miR treatment alone did not cause an apoptosis induction, their combination enhanced the apoptotic effect of prednisolone (Table 5, Figure 4, and Supplementary Figure 3). The combination of all anti-miRs and IC_50_ dose of prednisolone induced apoptosis 87.3 folds compared to the control group (*p* < 0.0001). Apoptosis induction was not detected in healthy B-lymphocytes (mean fold change 0.61, max. value 1.5, min. value 0.3, *p* > 0.05). Similar results were obtained from the JC-1 test which indicated mitochondrial membrane potential changes. Prednisolone treatment induced mitochondrial membrane potential change 13.10 folds compared to control in ALL cells (*p* < 0.0001; Table 6, Figure 5, Supplementary Figure 4). Alone anti-miR treatment did not cause a mitochondrial membrane potential change (only anti-miR-treated groups: fold change mean 2.60, *p* < 0.01); also, their combination did not enhance the prednisolone's effect (anti-miR and prednisolone combination groups: fold change mean 11.62, *p* < 0.01).

In addition, mitochondrial membrane potential change was not detected in healthy B-lymphocytes (mean fold change 1.37, max. value 1.6, min. value 0.8, *p* > 0.05).

## 4. Discussion

In this study, the anti-miR application was revealed to be effective on the viability, proliferation, cell cycle, and apoptosis of leukemia cells. In addition, this effect was increased with prednisolone administration, and this activity was found to be very low on healthy cells.

Since their discovery in the 1950s, glucocorticoids play an essential role in the treatment of ALL because of their ability to block cell-cycle progression and induce apoptosis in ALL cells. Many publications have reported a positive correlation between in vitro corticoid responses of leukemic lymphoblasts and in vivo responses to glucocorticoid monotherapy [11]. Among glucocorticoids, prednisolone has been the most commonly used drug in ALL therapy. It is already documented that there is significant interindividual variability in prednisolone sensitivity and early treatment response to glucocorticoid monotherapy is considered to be a strong prognostic factor [12–14]. These findings may be related to the leukemic cell prednisolone receptor affinity or postreceptor signaling pathways. Elucidation of these mechanisms that determines the relative cytotoxicity of prednisolone would help researchers to adjust precise dosing. For this reason, it is recommended to study the cytotoxicity of prednisolone to ALL cells before further applications [15]. Therefore, the IC_50_ value of prednisolone for the SUP-B15 cell line was determined as 20.20 *μ*M at the 48^th^ hour. Although there are studies including the prednisolone treatment in ALL cell lines, no IC_50_ concentration is determined. In the study conducted in 2011, Jiang et al. determined that the treatment of 1 *μ*g/ml to the SUP-B15 cell line decreased cell viability by 20% at the end of the 24^th^ hour and 80% at the end of the 48^th^ hour compared to the control group [9]. The cytotoxic effect of prednisolone on healthy B-lymphocytes was minimal; the IC_50_ dose was determined as 916.3 *μ*M at the 24^th^ hour for NCI-BL 2171 cells. In addition, there is no study in the literature showing the cytotoxic effect of prednisolone on NCI-BL 2171 cells.

The article "Antileukemic Effects of Anti-miR-146a, Anti-miR-155, Anti-miR-181a, and Prednisolone on Childhood Acute Lymphoblastic Leukemia" was retracted in 2024. Reasons: signs of a paper mill; compromised peer review; unreliable results or conclusions.

Currently, anti-miRNA-based therapy options are highly popular not only for offering the ability to regulate multiple genes but also for making a more cumulative effect on related proteins at different levels in the same pathway. Considering that cancer is a heterogeneous disease where various biological pathways get dysregulated; a single-agent therapy would not be sufficient, making miRNAs particularly valuable molecules. Research efforts on improving their specificity and efficacy for leukemia studies have been promoted as well [16].

Regarding prednisolone and miRNAs, there are few studies in the literature. In one study, it was shown that high levels of miR-128b and low levels of miR-223 show a significant correlation with good prednisolone response and better prognosis in childhood ALL [17] In another *in vitro* study, exogenous expression of miR-335 in leukemic cells was shown to increase the sensitization to prednisolone-mediated apoptosis and concluded that reintroducing miR-335 expression could be a promising therapeutic target for ALL treatment [18]. Additionally, Zhang et al. composed a set of miRNAs including miR-18a, miR-532, miR-218, miR-625, miR-193a, miR638, miR-550, and miR-633 and emphasized that these miRNAs can differentiate between a good or poor prednisone response in pediatric ALL [8].

Parallel to this data, it is already known that the expression levels of miR-146a, miR-155, and miR-181a are upregulated in ALL [9]. In line with the main purpose of the study, after determining the IC_50_ dose of prednisolone for cell lines, the cells were transfected with their relevant anti-miRs to investigate the molecular effects of silencing ALL-associated miRNAs and combining this silencing process with prednisolone treatment. Trypan blue viability test showed that each anti-miR administrations significantly reduced the viability of the cells. Although the viability of the anti-miR-155 group decreased by 45% compared to the control, the viability decreased below 50% in all other anti-miR-treated groups (anti-miR-146a 30%, anti-miR-181a 13%, and anti-let-7e 9% viability). As expected, the viability of the only prednisolone IC_50_-treated group is approximately 50% (41%). However, in all groups treated with anti-miR in combination with prednisolone, viability reduced below 15% (anti-miR-146a 2%, anti-miR-155 14%, anti-miR-181a 9%, and anti-let-7e 0% viability). Consistent with our findings, a recent study by Wang et al. stated that increased expression of miR-146a is an important factor in supporting cancer cell development in both childhood myeloid and lymphoid acute leukemias [19]. Likewise, El-Khazragy et al. suggested that the expression of miR-155 and miR-188a increased in ALL, and this increase in expression levels could be associated with poor prognosis [20]. On the other hand, studies are showing that the expression level of let-7e, which is a member of the let-7 miRNA group and defined as a tumor suppressor, is involved in the proliferation of healthy hematopoietic stem cells. It has been frequently documented to be downregulated in ALL patients [21]. However, in our study, it was determined that silencing of let-7e significantly reduced leukemia cell viability both alone and in combination with prednisolone groups. Although this seems to be contradictory to the previous literature, we anticipated that let-7e can regulate various signal pathways involved in the proliferation of ALL cells originating from hematopoietic stem cells.

The article "Antileukemic Effects of Anti-miR-146a, Anti-miR-155, Anti-miR-181a, and Prednisolone on Childhood Acute Lymphoblastic Leukemia" was retracted in 2024. Reasons: signs of a paper mill; compromised peer review; unreliable results or conclusions.

Silencing of all miRNAs, namely, miR-146a, miR-155, miR-181a, and let-7e in combination resulted in 14% viability. IC_50_ dose of prednisolone in addition to the combination group caused no viable cells to remain in this experimental group. There is no study in the literature involving the combinational silencing of these miRNAs together with prednisolone. Therefore, we believe that our results will contribute valuable insights regarding the molecular mechanisms of ALL.

According to the results of the APC-BrdU test, it was found that the treatments did not cause a significant change in the cell accumulation level in the G0/G1 and G2/M phases of SUP-B15 childhood ALL cells. However, the percentage of cells in the S phase has decreased significantly due to both prednisolone and anti-miR treatment. When compared to the control group, the number of cells in the treatment groups of anti-miR-146a, anti-miR-155, anti-miR-181a, anti-let-7e, and anti-miR combination in the S phase was decreased 66%, 58%, 71%, 32%, and 75%, respectively. The S phase accumulation decrease due to the anti-miR treatment correlates both with the results obtained from the viability tests and the findings obtained from the previously published studies [19, 20]. Prednisolone addition to anti-miR treatment groups caused the reduction in S phase accumulation by 92% on average (±4%). Consistent with the results achieved by Sloman and Bell, prednisolone treatment blocks the proliferation of ALL cells, especially during the transition of the cells to the S phase [22]. The G1/S checkpoint is a critical step in which DNA damage is checked before replication, DNA repair mechanism's function, and cells whose DNA damage cannot be repaired are directed to apoptosis [23]. The absence of significant changes in the G0/G1 phase of the cycle, but the dramatic decrease in accumulation in the S phase led us to comment that these applications forced most of the cells to apoptosis. It has been determined that prednisolone, anti-miR, and their combination did not cause a significant change in the cell cycle of NCI-BL 2171 healthy B-lymphocytes.

The article "Antileukemic Effects of Anti-miR-146a, Anti-miR-155, Anti-miR-181a, and Prednisolone on Childhood Acute Lymphoblastic Leukemia" was retracted in 2024. Reasons: signs of a paper mill; compromised peer review; unreliable results or conclusions.

Apoptotic effects of prednisolone, anti-miR, and their combination on the cells were evaluated using two different methods. According to the results of both Annexin V and JC-1 tests, prednisolone treatment significantly induced apoptosis of the SUP-B15 childhood ALL cells. Prednisolone treatment in combination with anti-miRs was determined to induce apoptosis at a higher rate in all groups than the mentioned anti-miR-alone-treated groups. Apoptosis induction was observed in all combination groups over 10-fold compared to the control. Strikingly, anti-miRs and prednisolone combination increased apoptosis 87.3-fold compared to control. Apoptosis induction was slightly increased in the anti-miR-only-treated groups. This can be explained by the fact that there are various overlapping points or cross-talks in the action mechanisms of those miRNAs. According to the results of Annexin V and JC-1 tests, it has been shown that application groups have no apoptotic effect on NCI-BL 2171 healthy B-lymphocytes. On the other hand, necrotic cell percentages in prednisolone treatment groups were determined as strikingly high compared to non-prednisolone-treated groups. Necrosis induction in different tissues, especially bone, is a common side effect of steroid-based drugs [24, 25].

## 5. Conclusions

The silencing of the critical leukemia regulatory miRNAs, namely, miR-146a, miR-155, and miR-181a may be regarded as an antileukemic strategy to enhance the effect of prednisolone treatment. Further studies involving different ALL cell lines and diverse miRNAs should be performed to reveal the potential effects and possible use of anti-miR agents in ALL therapy in the future.

The article "Antileukemic Effects of Anti-miR-146a, Anti-miR-155, Anti-miR-181a, and Prednisolone on Childhood Acute Lymphoblastic Leukemia" was retracted in 2024. Reasons: signs of a paper mill; compromised peer review; unreliable results or conclusions.

## Figures and Tables

**Figure 1:** Cytotoxic effects of prednisolone on (a) SUP-B15 and (b) NCI-BL 2171 cells.

**Figure 2:** Effects of anti-miR and prednisolone treatment on the viability of SUP-B15 and NCI-BL 2171 cells.

**Figure 3:** Cell cycle distribution of the treatment groups of (a) SUP-B15 and (b) NCI-BL 2171 cells.

**Figure 4:** Fold changes of the apoptotic cells compared to control (Annexin V).

**Figure 5:** Fold changes of the apoptotic cells compared to control (JC-1).

**Table 1:** Experimental groups.

Group #	Name	Group #	Name
1	Anti-miR-146a	7	Anti-miR-146a & IC_50_ dose of prednisolone
2	Anti-miR-155	8	Anti-miR-155 & IC_50_ dose of prednisolone
3	Anti-miR-181a	9	Anti-miR-181a & IC_50_ dose of prednisolone
4	Anti-let-7e	10	Anti-let-7e & IC_50_ dose of prednisolone
5	Anti-miR-146a + anti-miR-155 + anti-miR-181a combination	11	Anti-miR-146a + anti-miR-155 + anti-miR-181a combination & IC_50_ dose of prednisolone
6	Untreated control	12	IC_50_ dose of prednisolone

**Table 2:** Mature miRNA sequences.

miRNA	Sequence
hsa-miR-155-5p	UUAAUGCUAAUCGUGAUAGGGGUU
hsa-let-7a-5p	UGAGGUAGUAGGUUGUAUAGUU
hsa-miR-146a-3p	CCUCUGAAAUUCAGUUCUUCAG
hsa-miR-181a-3p	ACCAUCGACCGUUGAUUGUACC

**Table 3:** Effects of anti-miR and prednisolone treatment on the viability of SUP-B15 and NCI-BL 2171 cells.

Treatment group	Viability compared to control (%)		
	SUP-B15	NCI-BL 2171	
Anti-miR-146a	29.62^∗∗∗^	57.36	
Anti-miR-146a & IC_50_ dose of prednisolone	2.44^∗∗∗∗^	52.32	
Anti-miR-155	55.00	52.09	
Anti-miR-155 & IC_50_ dose of prednisolone	13.75^∗∗∗∗^	43.30	
Anti-miR-181a	13.03^∗∗∗∗^	58.18	
Anti-miR-181a & IC_50_ dose of prednisolone	9.17^∗∗∗∗^	46.91	
Anti-let-7e	9.17^∗∗∗∗^	49.82	
Anti-let-7e & IC_50_ dose of prednisolone	3.14^∗∗∗∗^	49.52	
Anti-miR-146a + anti-miR-155 + anti-miR-181a + anti-let-7e combination	13.75^∗∗∗∗^	41.10	
Anti-miR-146a + anti-miR-155 + anti-miR-181a + anti-let-7e combination & IC_50_ dose of prednisolone	0.00^∗∗∗∗^	52.22	
IC_50_ dose of prednisolone	41.25^∗^	56.91	

Fisher's exact test, *p*^∗^<0.05, ^∗∗∗^<0.001, and ^∗∗∗∗^<0.0001.

**Table 4:** Cell cycle distribution of the treatment groups on SUP-B15 and NCI-BL 2171 cells.

Treatment group	G_0_/G_1_ (%)		S (%)		G_2_/M (%)	
	SUP-B15	NCI-BL 2171	SUP-B15	NCI-BL 2171	SUP-B15	NCI-BL 2171
Anti-miR-146a	66.59	63.37	6.05	17.49	27.36	19.14
Anti-miR-146a & IC_50_ dose of prednisolone	74.23	52.36	3.09	26.18	22.68	21.46
Anti-miR-155	58.16	45.52	6.49	36.9	35.36^∗∗^	17.59
Anti-miR-155 & IC_50_ dose of prednisolone	75.30	73.29	1.22	4.82	23.48	21.89
Anti-miR-181a	74.85	67.87	6.44	15.9	18.71	16.23
Anti-miR-181a & IC_50_ dose of prednisolone	75.58	51.32	2.64	22.86	21.78	25.82
Anti-let-7e	58.85	52.67	11.96	25.35	29.19	21.98
Anti-let-7e & IC_50_ dose of prednisolone	49.68	38.14	0.65	29.66	49.68^∗∗^	32.20
Anti-miR-146a + anti-miR-155 + anti-miR-181a + anti-let-7e combination	66.50	72.90	4.40	9.92	29.10^∗^	17.18
Anti-miR-146a + anti-miR-155 + anti-miR-181a + anti-let-7e combination & IC_50_ dose of prednisolone	75.26	47.87	1.37	25.2	23.37	26.93
IC_50_ dose of prednisolone	55.21	55.67	0.47	19.15	44.31^∗∗^	25.18
Control	56.03	40.64	14.93	21.93	29.04	37.43

Fisher's exact test, *p*^∗^<0.05 and ^∗∗^<0.01.

The article "Antileukemic Effects of Anti-miR-146a, Anti-miR-155, Anti-miR-181a, and Prednisolone on Childhood Acute Lymphoblastic Leukemia" was retracted in 2024. Reasons: signs of a paper mill; compromised peer review; unreliable results or conclusions.

**Table 5:** Annexin V results of SUP-B15 and NCI-BL 2171 cells.

Treatment group	Live cell (%)		Necrotic cell (%)		Apoptotic cell (%)		Apoptotic fold change (to control)	
	SUP-B15	NCI-BL 2171	SUP-B15	NCI-BL 2171	SUP-B15	NCI-BL 2171	SUP-B15	NCI-BL 2171
Control	83.30	98.70	16.40	0.90	0.30	0.40	1.00	1.00
IC_50_ dose of prednisolone	5.70	97.30	84.60	2.20	9.70	0.60	32.30^∗∗∗∗^	1.50
Anti-miR-146a	76.20	96.80	23.40	2.80	0.30	0.40	1.00	1.00
Anti-miR-146a & IC_50_ dose of prednisolone	9.00	98.40	86.00	1.40	4.90	0.20	16.30^∗∗∗^	0.50
Anti-miR-155	80.70	94.00	15.80	5.40	3.60	0.60	12.00^∗∗^	1.50
Anti-miR-155 & IC_50_ dose of prednisolone	5.00	98.40	84.00	1.50	11.00	0.10	36.70^∗∗∗∗^	0.30
Anti-miR-181a	65.30	98.80	33.40	1.00	1.20	0.20	4.00	0.50
Anti-miR-181a & IC_50_ dose of prednisolone	4.10	98.70	81.20	1.20	14.70	0.00	49.00^∗∗∗∗^	0.00
Anti-let-7e	81.40	98.20	18.50	1.60	0.10	0.30	0.30	0.80
Anti-let-7e & IC_50_ dose of prednisolone	6.30	98.60	80.10	1.30	13.60	0.00	45.30^∗∗∗∗^	0.00
Anti-miR-146a + anti-miR-155 + anti-miR-181a + anti-let-7e combination	74.20	98.40	25.50	1.40	0.30	0.10	1.00	0.30
Anti-miR-146a + anti-miR-155 + anti-miR-181a + anti-let-7e combination & IC_50_ dose of prednisolone	5.60	98.50	68.10	1.40	26.20	0.10	87.30^∗∗∗∗^	0.30

Fisher's exact test, *p*^∗∗^<0.01, ^∗∗∗^<0.001, and ^∗∗∗∗^<0.0001.

**Table 6:** JC-1 results of SUP-B15 and NCI-BL 2171 cells.

Treatment group	Live cell (%)		Apoptotic cell (%)		Apoptotic fold change (to control)	
	SUP-B15	NCI-BL 2171	SUP-B15	NCI-BL 2171	SUP-B15	NCI-BL 2171
Control	92.30	74.10	7.60	20.90	1.00	1.00
IC_50_ dose of prednisolone	0.30	76.30	99.70	17.60	13.10^∗∗∗^	0.80
Anti-miR-146a	79.20	68.70	20.60	24.80	2.70	1.20
Anti-miR-146a & IC_50_ dose of prednisolone	5.40	47.10	94.50	43.40	12.40^∗∗^	2.10
Anti-miR-155	75.40	64.20	24.30	29.40	3.20	1.40
Anti-miR-155 & IC_50_ dose of prednisolone	16.20	49.80	83.80	40.10	11.00^∗∗^	1.90
Anti-miR-181a	86.20	73.10	13.70	21.30	1.80	1.00
Anti-miR-181a & IC_50_ dose of prednisolone	15.00	58.20	83.30	33.20	11.00^∗∗^	1.60
Anti-let-7e	80.00	69.50	19.20	23.10	2.50	1.10
Anti-let-7e & IC_50_ dose of prednisolone	16.00	59.70	84.00	31.70	11.10^∗∗^	1.50
Anti-miR-146a + anti-miR-155 + anti-miR-181a + anti-let-7e combination	79.90	72.50	19.80	20.90	2.60	1.00
Anti-miR-146a + anti-miR-155 + anti-miR-181a + anti-let-7e combination & IC_50_ dose of prednisolone	3.90	59.60	96.10	30.80	12.60^∗∗∗^	1.50

Fisher's exact test, *p*^∗∗^<0.01 and ^∗∗∗^<0.001.

The article "Antileukemic Effects of Anti-miR-146a, Anti-miR-155, Anti-miR-181a, and Prednisolone on Childhood Acute Lymphoblastic Leukemia" was retracted in 2024. Reasons: signs of a paper mill; compromised peer review; unreliable results or conclusions.

## Data Availability

The data is available on request from Bakiye Goker Bagca. Postal address: Aydin Adnan Menderes University, Faculty of Medicine, Department of Medical Biology, 09100, Aydin, Turkey. Email address: goker.bb@gmail.com.

## Supplementary Materials

Supplementary Materials Supplementary Figure 1: expression levels of SUP-B15 (a) and NCI-BL 2171 (b) cells. Supplementary Figure 2: cell cycle distribution of the treatment groups of SUP-B15 (a) and NCI-BL 2171 (b) cells. Supplementary Figure 3: Annexin V results of SUP-B15 (a) and NCI-BL 2171 (b) cells. Supplementary Figure 4: JC-1 results of SUP-B15 (a) and NCI-BL 2171 (b) cells.
